# The Nuance of Bilingualism as a Reserve Contributor: Conveying Research to the Broader Neuroscience Community

**DOI:** 10.3389/fpsyg.2022.909266

**Published:** 2022-06-24

**Authors:** Toms Voits, Vincent DeLuca, Jubin Abutalebi

**Affiliations:** ^1^PoLaR Lab, AcqVA Aurora Centre, UiT The Arctic University of Norway, Tromsø, Norway; ^2^Centre for Neurolinguistics and Psycholinguistics (CNPL), Vita-Salute San Raffaele University, Milan, Italy

**Keywords:** bilingualism, aging, reserve, resilience, dementia

## Abstract

The neurological notion of “reserve” arises from an individually observable dissociation between brain health and cognitive status. According to the cognitive reserve hypothesis, high-reserve individuals experience functional compensation for neural atrophy and, thus, are able to maintain relatively stable cognitive functioning with no or smaller-than-expected impairment. Several lifestyle factors such as regular physical exercise, adequate and balanced nutrition, and educational attainment have been widely reported to contribute to reserve and, thus, lead to more successful trajectories of cognitive aging (CA). In recent years, it has become clear that bilingualism is also a potential reserve contributor. Yet, there is little communication between the neuroscience of bilingualism research community and researchers working in the field of CA more generally, despite compelling reasons for it. In fact, bilingualism tends to be overlooked as a contributory factor in the CA literature, or reduced to a dichotomous trait, despite it being a complex experience. Herein, we discuss issues that are preventing recognition of bilingualism as a reserve contributor across all literatures, highlight the benefits of including language experiences as a factor of interest across research disciplines, and suggest a roadmap to better integrate bilingualism and aging moving forward. We close with calls toward a model of aging that examines the contributions across lifestyle factors, including that of bilingual experience.

## Introduction

Dementia is an umbrella term for a set of neurodegenerative diseases [of which Alzheimer’s disease (AD) is the most common one] with debilitating symptoms, primarily impairment of memory and other cognitive abilities, eventually leading to loss of autonomy over everyday activities. It is the leading cause of disability for older adults. Increased age is commonly (but not for all types of dementia) a risk factor for development of disease. As the average age of the global population increases, dementia is becoming an increased burden in both societal and financial terms around the world. Dementia was estimated to total to global annual costs of 1.3 trillion USD in 2019, and this figure is projected to reach between 1.7 and 2.8 trillion USD by 2030 (World Health Organization [WHO], 2021). Even in non-clinical aging, numerous cognitive processes and their neural underpinnings are known to naturally degrade (Fletcher et al., 2018; Salthouse, 2019). As there is currently no pharmacological cure of dementia, increasingly more interest has been devoted to understanding the factors that can help delay the onset of cognitive aging (CA) symptoms and promote the longevity of healthy life and cognition. Tackling dementia *via* preventive or treatment measures has thus been defined as a top societal and scientific priority (Winblad et al., 2016).

Given the absence of a cure, it is important to identify and study factors that contribute to cognitive resilience in healthy older individuals and people with dementia (Austad et al., 2019). Indeed, engagement in certain activities and lifestyle choices has been shown to lead to more successful CA outcomes (Harada et al., 2013). Bilingualism is one such component that holds promise as a lifestyle enrichment factor and a non-pharmacological contributor to delayed onset of dementia symptoms leading to preserved quality of life throughout aging. The effects of bilingualism on CA have been relatively widely reported in studies where language experiences themselves are of primary interest. Yet, it is seldom acknowledged in this capacity and often omitted from the relevant parallel literatures examining healthy and pathological aging from a clinical perspective. In other words, unlike other factors that are shown to affect neurocognitive outcomes in the older age, bilingualism is often overlooked. To illustrate this point, at the time of writing, a search for “bilingualism” and “aging” on PubMed returns only 344 results. This is in stark contrast to other lifestyle factors known to affect CA trajectories – for example “exercise” and “aging” yields 28,829 results, while “diet” and “aging” yields 25,480 results. The discrepancy between these figures clearly signals the perception of bilingualism as a factor of lesser interest in the context of understanding CA trajectories and outcomes. But why would that be? We submit that there are good reasons to consider bilingualism as part of a set of lifestyle experiences, known to affect CA and call for researchers across disciplines to consider including bilingualism as a covariate of interest moving forward. Collecting language background data across the wider neuroscientific domain (including clinical research) would help to capture some variance in the data that is currently left unaccounted for, while generating a wealth of language demographics of interest to bilingualism researchers. Herein, we discuss the need to convey bilingualism as a factor of interest to the broader neuroscience community and provide a roadmap for future directions in bilingualism and aging research.

## Reserve and Resilience

Cognitive aging is characterized by a marked decline across domains of cognition that can be observed starting from early adulthood (Salthouse, 2004). Nonetheless, there is individual variability in CA trajectories that becomes especially pronounced when facing neurodegeneration. As an example, AD pathophysiology is characterized by accumulation of abnormally folded amyloid-β peptide deposits or plaques in the brain, which are causally linked to further neurodegenerative processes (Scheltens et al., 2016). However, the correlation between amyloid burden on the brain and cognitive impairment is weak (Scarmeas and Stern, 2004). In fact, it is not uncommon to find amyloid deposits in the brains of people with no cognitive impairment at all (Aizenstein et al., 2008). This individual variability in cognitive outcomes in face of neural decline has been attributed to the notions of cognitive reserve (CR), brain reserve (BR), and brain maintenance (BM) (Stern, 2002; Stern et al., 2020).

The concepts of CR, BR, and BM have often been used to refer to similar and overlapping, yet diverse phenomena across different studies. To address this heterogeneity of terminology employed in the literature, a recently proposed consensus framework (Collaboratory on Research Definitions for Reserve and Resilience in Cognitive Aging and Dementia, 2022) suggests the following definitions. BR “reflects the neurobiological status of the brain at any point in time.” Those individuals who have greater BR from the outset, can tolerate more depletion before onset of any symptoms, i.e., BR translates to greater resilience against age- or disease-related structural atrophy over time. CR, on the other hand, is a theoretical concept that can be defined as a “property of the brain that allows for cognitive performance that is better than expected given the degree of life-course related brain changes and brain injury or disease.” As such, individuals who cognitively perform above expected for their levels of neural atrophy (or show no impairment at all, even with marked structural neural decline), are thought to exhibit high levels of CR. The framework also refers to BM, “the relative absence of changes in neural resources or neuropathologic change over time as a determinant of preserved cognition in older age.” As bilingualism has been argued to contribute to different types of reserve at different stages of life, and the exact relationship between BR, CR, and BM is unclear, we refer to improved CA outcomes as evidence for increases in *reserve* throughout the manuscript.

Previous research has identified many lifestyle predictors for greater reserve and more successful CA trajectories. These include occupational (Boots et al., 2015) and educational attainment (Mungas et al., 2018; Chan et al., 2021), sustained physical exercise (Sanchez-Lopez et al., 2018), healthy nutrition (Morris, 2012), increased social activity (Wilson et al., 2007), abstinence from smoking (Yaffe et al., 2009), general engagement in demanding cognitive activities (Wilson et al., 2021), and bilingualism (Bialystok et al., 2007; Bialystok, 2021). Reserve is built up over one’s lifetime, but continues to develop even in older age, where a combination of life experiences and lifestyle contribute to resilience against declines associated with aging (Burke et al., 2019). It has also been suggested that promoting reserve can be especially effective in populations that are genetically predisposed to dementia (Dekhtyar et al., 2019). Although there is plenty of evidence for reserve from epidemiological data, the neural basis of it is not as well understood (Steffener and Stern, 2012).

## Bilingualism as a Reserve Contributor

Why should bilingualism contribute to reserve? The answer to this question lies in the neurocognitive demands induced by managing two (or more) languages in the mind/brain. All available languages are activated in the bilingual or multilingual individual’s mind (Marian and Spivey, 2003). Therefore, bilingual language control requires engagement of cognitive control processes, so that the appropriate language is used in any given communicative context without undue interference of elements from any other languages. Given that all one’s languages maintain a level of activation at all times, bilingualism is a type of demanding cognitive activity that puts an extra strain on the brain and requires constant engagement of executive control and attentional resources (Bialystok and Craik, 2022). As the brain is a plastic organ that adapts to varied demands over time, the mental exercise of bilingual language control reinforces the brain structurally and affords stronger functional connectivity across the lifespan (Perani and Abutalebi, 2015). Indeed, there is currently over a decade’s worth of literature on neurocognitive adaptations in response to bilingualism, especially in aging populations where effects on CA trajectory and delayed onset of dementia/mild cognitive impairment (MCI) symptoms have been reported (see Gallo et al., 2022, for a recent review).

Literature to date seems to suggest that engagement with bilingual language use leads to a pattern of results corresponding with an interpretation of structural reserve (either BR or BM – in cross-sectional studies it is impossible to tell if structural differences observed are due to a greater initial baseline, a greater resilience to decay over time or, perhaps, a combination of both) in healthy older populations and a compensatory account of reserve (corresponding to the notion CR) in clinical populations, although the relationship is not always clear across different studies. In healthy aging populations bilinguals have been shown to have greater white matter volume (Olsen et al., 2015) and integrity (Luk et al., 2011; Anderson et al., 2018) across a variety of tracts and regions. In terms of gray matter, bilinguals, when compared to monolinguals, exhibit greater gray matter volume across anterior (Abutalebi et al., 2014), parietal (Abutalebi et al., 2015), temporal regions of the brain (Olsen et al., 2015), and the hippocampus (Voits et al., 2022). Evidence of structural reserve has also been found in bimodal bilinguals, showing that effects are not specific to spoken languages (Li et al., 2017). Any structural differences based on language groups seem to be on the account of better maintenance of existing structures over time (as opposed to growth of implicated areas) (Borsa et al., 2018; DeLuca and Voits, 2022), with a tendency for a more rapid decline in more advanced age, as this type of reserve gets exhausted (Heim et al., 2019). Functionally, older bilinguals exhibit greater neural efficiency by recruiting fewer neural resources than their monolingual counterparts to carry out a cognitive task (Gold et al., 2013; Anderson et al., 2021). Furthermore, language status has been shown to be a predictive factor in neural chemistry – bilingualism has been linked to a smaller concentration of AD biomarkers in cerebrospinal fluid, suggesting lower dementia risk in later life (Estanga et al., 2017), and metabolite concentration gradients in structures heavily implicated in cognitive control, which may potentially be a driving force for structural adaptations observed on a macroscopic scale (Pliatsikas et al., 2021).

Evidence for a compensatory account of reserve tends to manifest in studies where clinical aging populations are of interest whose brains have already been subject to structural decay. When matched on cognitive ability, bilingual individuals with AD show greater brain atrophy, suggestive of a compensatory reserve account (Schweizer et al., 2012; Duncan et al., 2018). Bilinguals also exhibit greater cerebral hypometabolism, cognitive performance being equal (Perani et al., 2017; Sala et al., 2022). Incidentally, when matched on brain health in older age where cognitive decline may occur, bilinguals seem to maintain their cognitive status, at a stage where some monolinguals start to exhibit symptoms of decline (Berkes et al., 2021). Taken together, this can be interpreted as bilinguals being able to compensate for neural tissue loss *via* potential formation of alternative neural networks or more efficient use of the resources available. In other words, bilinguals in either very advanced age or atypical aging are able to do more with less. Although the evidence presented so far on bilingualism and aging may seem contradictory at first glance, recent proposals suggest the accounts of bilingualism affecting BR and CR are in fact two different snapshots of the same overarching trajectory. In the first instance, BR manifests as preserved neural structure, whereas CR appears later and manifests as a dissociation between structure and cognition; specifically, preserved cognitive status despite accelerating neural decline (Bialystok, 2021). However, note that the relationship between and the neural basis of BR and CR is still not clear.

The first examination of bilingualism in connection with dementia symptom onset was a study investigating medical case records of monolingual and bilingual memory clinic patients, suggesting a 4-year later onset of dementia symptoms in bilingual individuals (Bialystok et al., 2007). This finding has been subsequently both supported (Craik et al., 2010; Clare et al., 2014; Woumans et al., 2015; Zheng et al., 2018) and contradicted (Yeung et al., 2014; Zahodne et al., 2014; Lawton et al., 2015) across various bilingual populations. Recent meta-analyses, however, have shown convincingly that bilingualism does indeed lead to a later expression of dementia symptoms, although the incidence is not affected by language status (Anderson et al., 2020; Brini et al., 2020; Paulavicius et al., 2020). Bilingualism effects appear independent of other confounders, such as education and migrant status (Alladi et al., 2013). Some studies have linked multilingualism (as opposed to bilingualism) to later symptom onset (Chertkow et al., 2010) and better cognition in healthy aging (Kavé et al., 2008), although bi- vs. multilingual effects remain under-researched.

Similar findings have been reported for MCI – where bilingualism has been found to delay symptom onset by as much as 7.4 years (Ramakrishnan et al., 2017; Calabria et al., 2020). More recently, a later onset of MCI symptoms followed by a more rapid decline and conversion to AD has been reported in bilinguals (Berkes et al., 2020). This finding is in line with the notion of a structural type of reserve, that, as the neural resources become exhausted, tips over to a more compensatory account. Finally, a population-level study revealed that countries where bilingualism was more prevalent reported lower incidence of dementia, lending further support to the notion of the protective nature of bilingualism on a much larger scale (albeit with less nuance) than any individual study can provide (Klein et al., 2016).

In addition to effects of MCI and AD, bilingualism has also been shown to correlate with less severe outcomes in acute neuropathology, such as stroke (Alladi et al., 2016; Paplikar et al., 2018). Moreover, it has been suggested to be a more general protective factor across other types of dementia where increases in reserve (*via* factors other than bilingualism) have been shown to lead to a more successful course of disease (Voits et al., 2020). Due to the mounting literature demonstrating bilingualism as a factor that leads to longer healthy aging and better cognitive outcomes in disease, bilingualism and language learning in the older age have been suggested as a viable public health strategy against CA and dementia (Bubbico et al., 2019), especially in low- and middle-income countries, where promoting reserve *via* other means can be difficult (Mendis et al., 2021).

Despite results showing bilingualism as a factor of interest, studies with otherwise comprehensive designs have omitted any mention of it completely. To provide some examples, Wirth et al. (2014) combined measures of education, cognitive activity, and physical activity with a set of biomarkers and related those to cognitive functioning and brain structure. However, bilingualism was not considered as a variable of interest. In a similar manner, Sowa et al. (2016) studied lifestyle and psychosocial patterns as predictors of healthy CA in Europe (where considerably more than half of the population can communicate in more than one language). While we applaud the consideration of many predictors of interest, the omission of language background and/or experience is a missed opportunity. As a final example, Darwish et al. (2018) examined links between education, occupational attainment, leisure activities and global cognitive functioning in an Arabic-speaking sample. In the demographic information, the authors report that 20.5% of participants spoke another language in addition to Arabic. Yet this factor was not included in statistical models, although, we maintain, it would be useful to see if it captures any of the variance in the data. While all the above are examples of well-conducted research, we aim to draw attention to the fact that they might have benefited from inclusion of a bilingualism measure and that future research should consider doing so, where possible. Bilingualism holds the promise of a significant reserve contributor factor and omitting this information is detrimental to the pursuit of better understanding the aggregate effects of lifestyle choices and experiences on CA outcomes.

Finally, although reserve (specifically CR) is often quantified *via* a proxy measure (years of education is a commonly used one) a set of CR measures have been developed over the years, in the form of self-reported questionnaires (Kartschmit et al., 2019). These tools are relatively quick and easy to administer and attempt to cover the life experiences and factors known to contribute to CR increases. However, in some cases, questions regarding individuals’ language background and experience are not included at all (e.g., CRIq; Nucci et al., 2012), or if they do, it is probed with a single question (e.g., CRQ, Rami et al., 2011; CRS, Leoñ et al., 2014). As we discuss below, this cannot provide sufficient richness of data to make any further inferences about the contributions of aspects of bilingualism that can lead to differential neurocognitive and health outcomes.

## A Complex Lifetime of Experiences

The picture painted above makes bilingualism appear an attractive lifestyle factor to investigate, not only within the remit of psychological and language sciences but also as a factor of interest in medical research, especially given the ubiquity with which language is used on a daily basis and across nearly every context in life. However, the diverse contexts and requirements for language use also entail a high degree of complexity in bilingual experience (see for Discussion, Titone and Tiv, 2022) and with it a potentially wide range of outcomes in terms of neurocognitive adaptations that would provide the basis for reserve accrual and deployment.

The complexity or degree of engagement in specific lifestyle factors is a widely accepted notion across other areas of aging research. Take, as an example, physical activity and the notion that it delays cognitive decline. It is not simply enough to practice once a week. In a longitudinal study Larson et al. (2006) followed cognitively normal older adults, and reported that those individuals who exercised three or more times per week were more likely to remain dementia-free during the 6-year follow-up period, independent of other risk factors. Likewise, Erickson et al. (2010) show that the amount of walking as a proxy of physical exercise was predictive of higher gray matter volume measured over a 9-year period. Specifically, walking more than 72 blocks/week was the threshold determined for protection against age-related changes in the hippocampus, prefrontal, and temporal brain regions. The amount of physical activity was also associated with a lower risk of developing MCI or dementia during the 9-year follow up. Translated to the bilingualism and neuroprotection field some parallels can be drawn: it should be the degree of second language engagement (usage, exposure, etc.) that provides the turning point. As outlined by Abutalebi et al. (2014) in a study on healthy bilingual seniors from Hong Kong, only those individuals who were still actively using their second language reported greater gray matter volumes in the temporal poles. Equally proficient bilinguals but with less engagement (i.e., usage of the second language) did not exhibit an equivalent level of neuroprotection.

A growing consensus in the field notes that bilingual language experience should not be reduced to a dichotomous distinction of “monolingual vs. bilingual” (just like physical activity should not be dichotomized as only “active vs. sedentary”). Rather it ought to be treated as a spectrum of experiences, where factors within bilingualism (such as age of acquisition, patterns and psychosocial contexts of language use, engagement and disengagement with languages over time) play a role and lead to differential adaptations in the brain (Green and Abutalebi, 2013; DeLuca et al., 2019, 2020; Beatty-Martínez et al., 2020; Pliatsikas, 2020; Gullifer et al., 2021). However, treating bilingualism as a continuous measure in research is relatively new in the field of bilingual neurocognition, and at present has only rarely been applied to aging. Several reasons may determine this. First, capturing and quantifying one’s bilingual experience is not a simple undertaking. At present, bilingualism is typically quantified as a composite of factor scores, based on self-reported language background and language use *via* questionnaires. Such questionnaires include the Language Experience and Proficiency Questionnaire (LEAP-Q; Marian et al., 2007), Language and Social Background Questionnaire (LSBQ; Anderson et al., 2018; see also Anderson et al., 2020 for a version applied specifically to aging), and Language History Questionnaire (LHQ3.0; Li et al., 2020). Moreover, recent evidence suggests that social context may both delineate these language experiences and have an impact on bilingualism-related neurocognitive outcomes in their own right (Bice and Kroll, 2019; Gullifer and Titone, 2020; Kałamała et al., 2021; Titone and Tiv, 2022).

It is clear that bilingualism is a complex lifetime of experiences. The bilingualism literature has shifted from a dichotomous, group-level analysis to one investigating individual differences by testing variables that make up one’s bilingual experiences and shows a gradient of neurocognitive adaptation commensurate with degree of experience (e.g., Kuhl et al., 2016; Gullifer et al., 2018; Sulpizio et al., 2020; Chung-Fat-Yim et al., 2021). Given the research showing the utility of an individual differences approach in young adults, it is prudent to contend with how these variations in bilingual experience might affect the trajectory of CA, particularly when juxtaposed against the variability within other lifestyle factors.

## Future Directions in Bilingualism and Aging Research

To summarize the above, research to date has shown bilingualism as a reserve contributor, although a truly interdisciplinary recognition of such findings has not come to be. We submit that this presents a limitation – to appreciate the effects of lifestyle choices and life experiences on CA more holistically, language background/experience should be considered alongside other reserve contributor factors and crucially in some nuance. While initial studies in the field bilingualism and neurocognition assessed bilingualism effects in absence of a more complete set of demographic, lifestyle, and background information as a necessary first step in this research program, it is imperative that nuanced information capturing individual variety across multiple domains of life gets collected moving forward. Equally, omitting bilingualism as a factor of interest does disservice to the pursuit of understanding individual variability in trajectories and outcomes of CA. This spans research focusing on both healthy aging and disease.

It can be argued that currently there is little interdisciplinary conversation between the bilingualism and the brain literature and the medical/neuroscientific community commonly concerned with aging research from a clinical perspective. Findings on bilingualism as a factor that has serious implications for CA outcomes primarily come from the former and tend to be published in linguistics, language sciences, and psychology journals that are seldom on the radar of medical professionals. This lack of connection/communication is something we hope will change moving forward.

To bridge this gap and solidify the status of bilingualism as a reserve contributor, research involving bilingualism needs to be conducted more akin to medical research. On the one hand this means starting collaborations with medical/neurological facilities and aging centers where typically studies on cognitive decline and dementia are carried out, and on the other, employing typical medical research protocols such as those that compare between different factors such as pharmacological studies and large-scale longitudinal studies similar to the Betula (Nilsson et al., 1997) or the Lothian Birth Cohort studies (Deary et al., 2007, 2012; see Bak et al., 2014, for a study focusing on bilingualism based on the Lothian Birth Cohort data). Similarly, large-scale population studies are also needed that would consider bilingualism together with other predictive factors and experiences. Studies based on already existing databases of neural and cognitive data can also be helpful [such as the Cambridge Centre for Ageing and Neuroscience (Cam-CAN) repository (Taylor et al., 2017)] provided future datasets like these have information on language experiences and bilingual language use patterns. A wealth of longitudinal data could also be collected with relative ease from patients as they present to memory clinics and even healthy individuals who may be invited to attend regular cognitive check-ups as they age and provide data on their language background and use. However, this is not an easy task for any individual research lab. Coordination and multi-lab collaborations would allow for not only capturing diversity of language contexts but also be helpful in identifying any possible interaction of language use by context on aging (for a roadmap on multi-lab collaborations, see Leivada et al., 2021). Finally, such collaborations would also provide adequate sampling power to more robustly test the effects of multiple complex life experiences on CA trajectories.

A key factor to consider, however, is the operationalization and quantification of bilingual experiences moving forward. One needs to be mindful of the fact that bilingualism is a multifaceted and multidimensional life experience that can be difficult to gauge and quantify, yet future research should embrace this complexity in a responsible manner. We need to move beyond asking simplistic questions that lead to a false dichotomous collapsing across groups and find a way to address the complexity of language experience. Large datasets alone cannot act as a substitute for detailed data that acknowledges the complexity of bilingual experience (see, e.g., Nichols et al., 2020). However, one needs to consider the practicality for including lengthy questionnaires tapping in language experiences in medical practice. By definition, it will need to be a balancing act between attempts to capture as much variance and detail as possible, and the practical feasibility of implementing such tools.

To note, collecting language background information is important not only for those who self-identify as bilinguals, but also those who consider themselves monolingual – as variability in exposure to foreign languages and dialects can be observed even within this group (Castro et al., 2022) and passive language experiences can have observable effects on brain function (Bice and Kroll, 2019; Bice et al., 2020). There is variability even in the monolingual end of the -lingualism spectrum that may be deterministic for CA trajectories.

Finally, the most straight-forward way ahead at present is to conduct comparative studies where bilingual experiences are evaluated in the context of one’s wider life experiences and lifestyle choices. And thus, a well-designed study would test one’s linguistic background and language use patterns across the lifespan but do so together with information about other factors that are known to contribute to differential outcomes in older age. In essence, future research should try to build complex individual neurocognitive profiles to tease apart individual contributions of reserve contributor factors. Such combined datasets would afford the evaluation of one’s cognitive status, structural/functional brain health and also provide insights on the individual and combined effects of bilingualism and other reserve contributor factors.

To conclude, bilingual language experiences have already been shown to affect the mind and brain, across the lifespan and in older populations. It is now essential to work toward solidifying bilingualism (as the multidimensional, rich set of experiences that it is) as a factor of interest in the CA/medical field and clearly communicate findings of bilingualism as a reserve contributor to the medical and clinical aging literatures. Future research needs to measure and quantify individual language experiences and test what language use behaviors and practices contribute most to successful CA outcomes, while also being mindful of the fact that bilingualism is one of several predictive experiences of one’s lifetime.

## Data Availability Statement

The original contributions presented in this study are included in the article/supplementary material, further inquiries can be directed to the corresponding author.

## Author Contributions

TV, VD, and JA contributed to the conception of the manuscript. TV wrote the first draft of the manuscript. VD and JA wrote sections of the manuscript. All authors contributed to the manuscript revision, read, and approved the submitted version.

## Conflict of Interest

The authors declare that the research was conducted in the absence of any commercial or financial relationships that could be construed as a potential conflict of interest.

## Publisher’s Note

All claims expressed in this article are solely those of the authors and do not necessarily represent those of their affiliated organizations, or those of the publisher, the editors and the reviewers. Any product that may be evaluated in this article, or claim that may be made by its manufacturer, is not guaranteed or endorsed by the publisher.
